The article "XBP1 inhibits mesangial cell apoptosis in response to oxidative stress via the PTEN/AKT pathway in diabetic nephropathy" was retracted in 2024. Reasons: duplicated images; unreliable results or conclusions.

# XBP1 inhibits mesangial cell apoptosis in response to oxidative stress via the PTEN/AKT pathway in diabetic nephropathy

**DOI:** 10.1002/2211-5463.12655

**Published:** 2019-06-02

**Authors:** Yan Wang, Zhong He, Qiu Yang, Guangju Zhou

**Affiliations:** ^1^ Department of Endocrinology the Affiliated Hospital of North Sichuan Medical College Nanchong China; ^2^ Institute of Basic Medicine North Sichuan Medical College Nanchong China

**Keywords:** apoptosis, mesangial cell, oxidative stress, PTEN/AKT pathway, XBP1

## Abstract

Diabetic nephropathy (DN) is a complication of diabetes mellitus (DM) that frequently results in renal disease, and is characterized by a variety of symptoms, including albuminuria. It has been shown that apoptosis of glomerular mesangial cells (MCs) can aggravate albuminuria and contribute to the development of diabetic glomerulosclerosis. Hence, determination of the mechanisms leading to MC apoptosis may help us gain insights into the pathogenesis of DN. As our understanding of the role of high glucose (HG) in MC apoptosis remains elusive, we explored the interplay between X‐box binding protein 1 (XBP1) and MC apoptosis in this study. XBP1 was observed to be downregulated both *in vivo* and *in vitro*. Treatment of XBP1‐overexpressing cells with HG resulted in a decrease of reactive oxygen species (ROS) and a suppression of cell apoptosis, concomitant with decreases in cleaved caspase‐3 and Bax. Subsequent analyses demonstrated that XBP1 overexpression inhibited the expression of phosphatase and tensin homolog deleted on chromosome ten (PTEN) and enhanced the activation of AKT in MCs exposed to HG. In addition, XBP1‐induced injuries in MC were reversed by overexpression of PTEN, and XBP1 inhibited apoptosis, which was mediated by the activated PTEN/AKT signaling pathway. Thus, our data indicate that XBP1 can activate the PTEN/AKT signaling pathway, thereby alleviating oxidative stress caused by HG or MC apoptosis. These findings suggest that XBP1 may have potential in the development of treatment methods for DN.

**Abbreviations**
DM: diabetes mellitus
DMEM: Dulbecco's modified Eagle's medium
DN: diabetic nephropathy
ER: endoplasmic reticulum
HG: high glucose
MCs: mesangial cells
PI: propidium iodide
PTEN: phosphatase and tensin homolog
ROS: reactive oxygen species
XBP1: X‐box binding protein 1

## Introduction

Diabetic nephropathy (DN) is a complication of diabetes mellitus (DM) that frequently results in renal disease 1. Clinically, DN is characterized by a variety of symptoms such as albuminuria 2. Many patients have progressive renal injury 3, 4, despite the rapid development of therapies for DN 5, 6, 7. Thus, it is of priority to develop more efficient methods to delay or reverse the progression of DN.

The article "XBP1 inhibits mesangial cell apoptosis in response to oxidative stress via the PTEN/AKT pathway in diabetic nephropathy" was retracted in 2024. Reasons: duplicated images; unreliable results or conclusions.

It has been recognized that glomerular mesangial cells (MCs) are involved in a variety of events and play critical roles 8, 9. Increasing evidence has confirmed that MC apoptosis contributes to the aggravation of albuminuria and the development of diabetic glomerulosclerosis, which shows a close correlation with DN 10, 11, 12. Hence, determination of the possible mechanism that leads to MC apoptosis can help us gain insights into the pathogenesis of DN.

It has been commonly recognized that reactive oxygen species (ROS) are key factors that mediate a series of biological events, including apoptosis 13, and previous studies have shown that ROS have a critical role in the development of DN 14, 15, 16. Moreover, *in vivo* and *in vitro* evidence has demonstrated that ROS initiate the dysfunction of MCs first, followed by the apoptotic program, which further triggers altered homeostasis and the development of DN 17, 18.

X‐box binding protein 1 (XBP1), a critical regulator of endoplasmic reticulum (ER) stress 19, is altered in DN progression 20. Furthermore, it has been suggested that XBP1 can prevent oxidative stress 21. Despite its protective role against ER stress, the mechanisms of action of XBP1 remain elusive.

In this study, we analyzed the expression profile of XBP1 in renal tissue samples and detected how XBP1 protected MCs against the effects of high glucose (HG)‐induced ROS and apoptosis. We investigated the involvement of the phosphatase and tensin homolog (PTEN)/AKT signaling pathway in the protective effects of XBP1. We showed that XBP1 is a possible indicator for the diagnosis and treatment of DN.

## Materials and methods

### Animals

C57BL/6 mice and db/db mice were provided by Experimental Animal Center of North Sichuan Medical College and maintained at a controlled temperature (22–23 °C, 55% ± 5% humidity). The mice had free access to food and water. All animal procedures were approved by the Animal Experimentation Ethics Committee of the Affiliated Hospital of North Sichuan Medical College.

### Cell culture

A rat MC line HBZF‐1 (CCTCC, Wuhan, China) was cultured in Dulbecco's modified Eagle's medium (DMEM) 22. To the DMEM, penicillin, streptomycin, 10% FBS, and glucose were also added. Prior to HG treatment, confluent cells were transferred to serum‐free DMEM for overnight incubation.

### Quantitative reverse transcription PCR

Total RNA was extracted from cells and samples using TRIzol^®^ reagent (Invitrogen, Carlsbad, CA, USA; Thermo Fisher Scientific, Inc., Waltham, MA, USA) according to the manufacturer's protocol and subsequently purified with the RNeasy Mini Kit (Qiagen GmbH, Hilden, Germany). Reverse transcription was performed with PrimeScript^™^ 1st Strand cDNA Synthesis Kit (Takara) according to standard protocol. Quantitative real‐time PCR was performed on an ABI 7300 Real‐Time PCR System ( Applied Biosystems, Osaka, Japan) using the Fast Start Universal SYBR Green Master (Rox) (Roche Diagnostics Ltd., Shanghai, China). PCR thermal cycle parameter settings were as follows: 95 °C for 10 min, 40 cycles at 60 °C for 60 s, and 95 °C for 15 s, followed by a melting curve from 60 °C to 95 °C to ensure amplification of a single amplification product. Glyceraldehyde‐3‐phosphate dehydrogenase (GAPDH) was used as an endogenous control. Fold changes were calculated using the 2^‐ΔΔCq^ method. In this experiment, the following primer sequences were synthesized by Sangon Biotech Co., Ltd (Shanghai, China): XBP1 forward: 5′‐TTACGAGAGAAAACTCATGGGC‐3′; XBP1 reverse: 5′‐ACACATAGCGCCTCTGACTG‐3′; GAPDH forward: 5′‐GGGTCCAACTTGTCCAGAATGC‐3′; and GAPDH reverse: 5′‐AGAAGGCTGGGGCTCATTTG‐3′. Experiments were conducted in triplicate.

The article "XBP1 inhibits mesangial cell apoptosis in response to oxidative stress via the PTEN/AKT pathway in diabetic nephropathy" was retracted in 2024. Reasons: duplicated images; unreliable results or conclusions.

### Transfection

To express PTEN and XBP1 in HBZF‐1 cells, we utilized pcDNA‐PTEN and XBP1 (Shanghai GeneChem Co., Ltd., Shanghai, China) to transfect the cells, and an empty vector was used as the control. To reduce the XBP1 expression in HBZF‐1 cells, we utilized XBP1‐specific siRNA (si‐XBP1) (Shanghai GeneChem Co., Ltd.) to transfect the cells, and negative control (si‐Con) was used as the control. HBZF‐1 cells were transfected using Lipofectamine 2000 (Invitrogen), following the manufacturer's protocol. Transfection admixture was generated via deliquating 4μg of plasmid DNA as well as 3μL of Turbofect reagent (Fermentas, Glen Burnie, MD, USA) in 500 μL of DMEM/F12 medium without serum, via tender pipetting. Following incubation for 20 minutes, the transfection mixture was added to the culture medium and incubated for 24 h and then treated with HG for 24 h.

### Evaluation of cell apoptosis

Flow cytometry was performed to evaluate cell death. The obtained cells were washed twice with cold PBS and subsequently centrifuged for 5 min at 100 rpm, after which the supernatant was discarded. The pellet was resuspended in binding buffer. Following 10 min of incubation with a mixture of propidium iodide (PI) and FITC‐Annexin V, the fluorescence signals were assessed.

### Measurement of intracellular ROS

Cells were incubated in the presence of 25 μm H2 DCF‐DA for 30 min and then washed twice with PBS. The fluorescence intensity at 515 nm excitation wavelength and 585 nm emission wavelength was measured using a luminometer (Tecan, Salzburg, Austria). In this experiment, the intensity of ROS generation in cells without any treatment was regarded as 100%.

The article "XBP1 inhibits mesangial cell apoptosis in response to oxidative stress via the PTEN/AKT pathway in diabetic nephropathy" was retracted in 2024. Reasons: duplicated images; unreliable results or conclusions.

### Assay of superoxide dismutase (SOD1) activity

All used reagents were purchased from Sigma‐Aldrich Sp. z o.o. (Poznań): (‐) epinephrine, HCl, 0.05 M Na_2_CO_3_/NaHCO_3_ buffer (pH 10.2), EDTA‐Na2, chloroform, ethanol—and were used to SOD extraction. In a test tube, a mixture of hemolysate, chloroform, and ethanol solution (3:5; v/v) and distillated water were combined. Afterward, the mixture was energetically vortexed and centrifuged (5 min; 4 °C; 3824 g). Next to the SOD extract, the Na2CO3/NaHCO3 buffer and adrenaline were added and the mixture was incubated for three min at 37 °C. The analysis of SOD1 activity was performed using a UV/VIS Lambda 40 spectrophotometer (PerkinElmer, New York, NY, USA). The analysis of the study materials’ absorbency was performed over five min at a wavelength of 320 nm (at 30 °C). SOD1 activity was calculated per 1 g of RBC hemoglobin. Sensitivity of the assay was 0.1 U·mL^−1^, specificity 97%, while coefficient of variation was lower than 4%.

### Assay of catalase (CAT) activity

Reagents (50 mm phosphoric buffer, pH 7.0 (KH2PO4, Na2HPO4x12 H2O), H2O230 mm) were purchased from Sigma‐Aldrich Sp. z o.o. (Poznań). Hemolysate was diluted 500‐fold using a 50 mm phosphoric buffer. Catalase activity was analyzed using a UV/VIS Lambda 40 spectrophotometer (PerkinElmer). Absorbance measurements of the study sample (hemolysate and 30 mm H2O2 solution) were performed within 30 sec at a wavelength of 1240 nm (at 30 °C). Catalase activity was determined based on the calibration curve, obtained as a result of assays performed for several solutions of the catalase activity pattern (Oxis Research, Foster, CA, USA). Catalase activity was calculated per 1 g of the erythrocytes’ hemoglobin. Sensitivity of the assay was 1.71 U·mL^−1^, specificity 89%, while coefficient of variation was lower than 2%.

### Western blotting analysis

Homogenization was carried out using NP‐40 lysis buffer (Beyotime, China). Proteins were separated via SDS/PAGE and transferred to a PVDF membrane (Millipore, MA, USA). The membrane was blocked with 5% BSA for 1 h at room temperature. Proteins were probed with anti‐XBP1, anti‐Bax, anti‐PTEN, anti‐p‐AKT, anti‐AKT, and anti‐β‐actin antibodies (Cell Signaling Technology, Waltham, MA, USA) for 12 h at 4 °C. Following 4 washes in Tris‐buffered saline supplemented with Tween‐20 (TBST), immunoblots were detected with a secondary antibody conjugated to HRP. The bands were developed using a chemiluminescence reagent (Pierce, IL, USA). The protein bands were analyzed using the Omega 16ic Chemiluminescence Imaging System software (version 17; Ultra‐Lum, Inc., Claremont, CA, USA). The relative protein level was normalized by the intensity of b‐actin, and the averaged relative protein level in control group is defined as 1.0.

The article "XBP1 inhibits mesangial cell apoptosis in response to oxidative stress via the PTEN/AKT pathway in diabetic nephropathy" was retracted in 2024. Reasons: duplicated images; unreliable results or conclusions.

### Statistics

Data, in the form of the mean ± SEM, were compared between groups using a two‐tailed, unequal‐variance Student's *t*‐test, or ANOVA, followed by Tukey's post hoc analysis. *P* < 0.05 was indicative of a statistically significant difference.

## Results

### XBP1 is downregulated in diabetic mouse glomeruli and in MCs exposed to HG

To explore the role of XBP1 in DN, real‐time PCR of XBP1 was performed using glomeruli from db/db mice and MCs treated with HG *in vitro*. XBP1 was significantly reduced in the glomeruli from db/db mice compared with that in the glomeruli from wild‐type (WT) mice (Fig. 1A–**C**). Similarly, XBP1 was downregulated in the MCs treated with HG compared with the control level (Fig.**** 1D). Moreover, the protein level of XBP1 was lower in db/db mice and in the MCs following treatment with HG than in the control. In addition, the expression of PTEN was significantly increased and the expression of p‐AKT was significantly decreased in the glomeruli from db/db mice compared with that in the tissue from WT mice (Fig. 1E,F).

**Figure 1:** X‐box binding protein 1 is downregulated in diabetic mouse glomeruli and in MCs exposed to HG. (A,B) Decreased expression of XBP1 in db/db mouse glomeruli (A) and in MCs treated with HG (B), as determined by quantitative reverse transcription PCR (qRT/PCR). (C,D) Decreased expression of XBP1 in db/db mouse glomeruli (C) and in MCs treated with HG (D), as determined by western blotting. (E,F) Decreased expression of p‐AKT (E) and increased expression of PTEN (F) in db/db mouse glomeruli (C) and in MCs treated with HG (D), as determined by western blotting. Data are represented as the mean ± SEM. The experiment was conducted in triplicate. **P < 0.01 vs. the control group. (unpaired *t*‐test).

### XBP1 suppresses oxidative stress in HG‐treated MCs

Oxidative stress is a crucial factor for the development of DN 23. An evident increase in ROS levels was observed in HG‐treated cells; the values were significantly higher than that for their counterparts (Fig. 2A,B). However, a reverse trend was observed in the presence of overexpressed XBP1. Moreover, XBP1 overexpression markedly increased SOD1 and CAT levels compared to the vector control (Fig. 2C,D). In addition, XBP1 knockdown significantly increased the HG‐induced ROS production and reduced the level of SOD1 (Fig. 2E,F). These results demonstrated that XBP1 suppresses ROS overproduction in MCs under diabetic conditions.

**Figure 2:** X‐box binding protein 1 suppresses HG‐induced oxidative stress in MCs. After 24 h of transfection with an XBP1 plasmid (XBP1) or empty vector (vector), MCs were treated with HG for 48 h. (A) Intracellular generation of ROS by transforming H2DCF‐DA to DCF via an oxidative reaction. Scale bars: 100 μm. (B) Quantification data for the ROS level of each group. (C) SOD1 activity detection. (D) CAT activity detection. After 24 h of transfection with XBP1‐specific siRNA (si‐XBP1) or negative control (si‐Con), MCs were treated with HG for 48 h. (E) Quantification data for the ROS level of each group. (F) SOD1 activity detection. Data are represented as the mean ± SEM. The experiment was conducted in triplicate. **P < 0.01 vs. the control group; ^#^ *P* < 0.05 vs. the vector + HG group or the si‐Con + HG group. One‐way ANOVA with Tukey's post hoc test.

The article "XBP1 inhibits mesangial cell apoptosis in response to oxidative stress via the PTEN/AKT pathway in diabetic nephropathy" was retracted in 2024. Reasons: duplicated images; unreliable results or conclusions.

### XBP1 attenuates HG‐induced MC apoptosis

The induction of oxidative stress is an important mechanism that underlies HG‐induced MC apoptosis 24. Thus, we attempted to determine how ROS regulate the effects of XBP1 on apoptosis. As shown in Fig. 3A,B, apoptosis was observed in HBZF‐1 cells after HG treatment, which was inhibited after the induction of XBP1 overexpression. Bax and cleaved caspase‐3, which are indicators of apoptosis, were upregulated in HG‐treated cells compared with that in normal cells. Similarly, after overexpression of XBP1, Bax and cleaved caspase‐3 were downregulated (Fig. 3C–E). In contrast, XBP1 knockdown significantly increased the MC apoptosis induced by HG treatment (Fig. 3F).

**Figure 3:** X‐box binding protein 1 attenuates HG‐induced cell apoptosis in MCs. After 24 h of transfection with an XBP1 plasmid (XBP1) or empty vector (vector), MCs were treated with HG for 48 h. (A) Representative image of cell apoptosis determined via flow cytometry. (B) Quantification data for the apoptotic cells for each group. (C–E) Representative immunoblots (C) and quantitative analysis of Bax (D) and cleaved caspase‐3 (E) in MCs. After 24 h of transfection with XBP1‐specific siRNA (si‐XBP1) or negative control (si‐Con), MCs were treated with HG for 48 h. (F) Quantification data for the apoptotic cells for each group. Data are represented as the mean ± SEM. The experiment was conducted in triplicate. **P < 0.01 vs. the control group; ^#^ *P* < 0.05 vs. the vector + HG group or the si‐Con + HG group. One‐way ANOVA with Tukey's post hoc test.

### XBP1 activates the AKT signaling pathway through downregulation of PTEN in MCs

We screened the signaling pathways involved in the XBP1‐mediated injury of MCs in the presence of HG. Considering that the PTEN/AKT signaling pathway is critical for oxidative stress and apoptosis 25, we aimed to determine how XBP1 activates the PTEN/AKT signaling pathway in HBZF‐1 cells treated with HG. The results showed that in addition to a remarkable increase in PTEN, the phosphorylation of AKT decreased inHBZF‐1 cells with HG‐induced injuries compared with that in cells treated with normal glucose (Fig. 4A–D). We transfected the HG‐treated HBZF‐1 cells with plasmids to overexpress XBP1 and found that PTEN was downregulated with an increase in the expression of phosphorylated AKT, but with no alteration in the total AKT.

The article "XBP1 inhibits mesangial cell apoptosis in response to oxidative stress via the PTEN/AKT pathway in diabetic nephropathy" was retracted in 2024. Reasons: duplicated images; unreliable results or conclusions.

**Figure 4:** X‐box binding protein 1 activates the AKT signaling pathway through downregulation of PTEN in MCs. After 24 h of transfection with an XBP1 plasmid (XBP1) or empty vector (vector), MCs were treated with HG for 48 h. A–D**,** Representative immunoblots (A) and quantitative analysis of PTEN (B), phosphorylation of AKT (C), and total AKT (D) in MCs. Data are represented as the mean ± SEM. The experiment was conducted in triplicate. **P < 0.01 vs. the control group; ^#^ *P* < 0.05 vs. the vector+HG group. One‐way ANOVA with Tukey's post hoc test.

### PTEN/AKT signaling pathway is critical for the protective effect of XBP1 against oxidative stress and apoptosis

To determine whether the downregulation of PTEN contributes to the antagonistic effect of XBP1 against the apoptosis induced by HG treatment, we transfected HBZF‐1 cells with plasmids to overexpress PTEN. The results indicated that PTEN overexpression abolished the reduction of ROS generation and the suppression of apoptosis (Fig. 5A–E).

**Figure 5:** The PTEN/AKT signaling pathway is significant in mediating the protective effect of XBP1 against oxidative stress and apoptosis. After 24 h of cotransfection with an XBP1 plasmid (XBP1) or PTEN plasmid (PTEN), MCs were treated with HG for 48 h. (A) Intracellular generation of ROS by transforming H2DCF‐DA to DCF via an oxidative reaction. (B) SOD1 activity detection. **(**C) CAT activity detection. (D–E) Representative of cell apoptosis by flow cytometry. Data are represented as the mean ± SEM. The experiment was conducted in triplicate. **P < 0.01 vs. the control group; ^#^ *P* < 0.05 vs. the HG group; ^$^ *P* < 0.05 vs. the XBP1+HG group. One‐way ANOVA with Tukey's post hoc test.

## Discussion

In this study, we clarified that XBP1 is significantly downregulated in DN mice, while overexpression of XBP1 can abolish HG‐induced apoptosis in HBZF‐1 cells with a reduction in ROS generation. The most important finding is the involvement of the PTEN/AKT signaling pathway in mediating the antagonistic effect of XBP1 on increased apoptosis and ROS generation, induced by HG treatment, suggesting that XBP1, together with PTEN/AKT, comprises a novel axis, which is a novel target for the development of new methods for DN treatment.

The article "XBP1 inhibits mesangial cell apoptosis in response to oxidative stress via the PTEN/AKT pathway in diabetic nephropathy" was retracted in 2024. Reasons: duplicated images; unreliable results or conclusions.

Currently, as the most frequent complication of DM 26, DN has been found in 40% or more of the novel DM cases 15. Nevertheless, information regarding DN‐associated pathogens remains elusive. Studies on DM‐related renal injuries have shown the role of oxidative stress in the development and progression of DN 27. An increase in ROS is correlated with a variety of factors, for example, renal epithelial dysfunction 28. XBP1 is associated with the synthesis of multiple proteins and pathological processes 29. It exists in a variety of human tissues, including the kidney 30. XBP1 has been shown to be involved in a series of biological events, such as cardiac myogenesis 31, and its activation is mediated by post‐transcriptional modifications 32. In this study, we found that XBP1 was downregulated in kidney tissues from db/db mice and in MCs treated with HG, suggestive of a potential correlation between XBP1 and DN.

The central roles of MCs in the glomerulus have been clarified in a variety of studies. In addition to maintaining the capillary loop, MCs are also involved in mediating the apoptotic activity of multiple cells 33. Nephrons are conventionally believed to be the units that comprise the structural and functional basis of the kidney, and decreased nephrons can cause proteinuria by damaging glomerular filtration and reabsorption by renal tubules 34. As DN progresses into the mid‐ or late‐stage, cellular apoptosis increases in the glomerulus, leading to a destructive effect on glomerular filtration, which further aggravates the albuminuria 35. The apoptotic activity of MCs is critical for the development of glomerulosclerosis, which has been considered to be a contributing factor for ESRD 36. Additionally, oxidative stress has been found to have a crucial role in DN 37. In HG‐treated MCs, NADPH oxidase is overactivated and ROS are excessively generated, which may result in MC apoptosis 38. In contrast, normalization of oxidative stress using antioxidants reduces the MC injury in diabetes 18. In the present study, overexpression of XBP1 decreased HG‐induced ROS generation and apoptosis of MCs, suggesting that XBP1 may block the progression of DN, as demonstrated by the antagonistic effects against apoptosis and oxidation.

In addition to the consensus that PTEN has a pro‐apoptotic role, previous studies have reported the critical role of PTEN in DM, as well as its complications 39. PTEN downregulation has been found to be related to hypertrophy in a hyperglycemic model of MCs 40. Additionally, in the liver or fat tissues of db/db mice, PTEN downregulation can prevent the development of DM 41. Furthermore, it has been demonstrated that the PTEN/AKT signaling pathway is associated with the modulation of various biological events, including the development of DN. The alleviating effects of notoginsenoside R1 (NR1) against the kidney injuries of DN mice have been reported, which have been confirmed by the activation of the AKT signaling pathway 42. Additionally, after the administration of Jiang tang decoction, KK‐Ay mice exhibited a significant reduction of DN‐related inflammatory responses with upregulation of the PTEN/AKT signaling pathway 43. In the presence of miR‐25, the PTEN/AKT signaling pathway is altered in HepG2 cells 44. In this study, we screened the possible pathways through which XBP1 modulates HG‐induced apoptosis. Overexpression of XBP1 upregulated p‐AKT (Ser473) with a decrease in PTEN in the MCs treated with HG. More importantly, the inhibitory effects of XBP1 against HG‐induced ROS generation and apoptosis were reversed by the overexpression of PTEN. Thus, the involvement of XBP1 in HG‐induced MC apoptosis is realized based on the PTEN/AKT pathway, implicating a critical role for the XBP1/PTEN/AKT axis in DN.

The article "XBP1 inhibits mesangial cell apoptosis in response to oxidative stress via the PTEN/AKT pathway in diabetic nephropathy" was retracted in 2024. Reasons: duplicated images; unreliable results or conclusions.

## Conclusions

Taken together, XBP1 is downregulated in DN. Increased ROS generation and apoptotic activity in the MCs treated with HG can be suppressed by the overexpression of XBP1. Thus, XBP1 serves as a possible target for the development of treatment strategies for DN.

## Conflict of interest

The authors declare no conflict of interest.

## Author contributions

In this work, YW and GZ conceived the study and designed the experiments. ZH and QY contributed to the data collection, performed the data analysis, and interpreted the results. YW wrote the manuscript. GZ contributed to the critical revision of article. All authors read and approved the final manuscript.
